# Application of Machine Learning to Predict Estimated Ultimate Recovery for Multistage Hydraulically Fractured Wells in Niobrara Shale Formation

**DOI:** 10.1155/2022/7084514

**Published:** 2022-06-21

**Authors:** Ahmed Farid Ibrahim, Sulaiman A Alarifi, Salaheldin Elkatatny

**Affiliations:** ^1^Department of Petroleum Engineering and Geosciences, King Fahd University of Petroleum & Minerals, Dhahran 31261, Saudi Arabia; ^2^Center for Integrative Petroleum Research, King Fahd University of Petroleum & Minerals, Dhahran 31261, Saudi Arabia

## Abstract

The completion design of multistage hydraulic fractured wells including the cluster spacing injected proppant and slurry volumes has shown a great influence on the well production rates and estimated ultimate recovery (EUR). EUR estimation is a critical process to evaluate the well profitability. This study proposes the use of different machine learning techniques to predict the EUR as a function of the completion design including the lateral length, the number of stages, the total injected proppant and slurry volumes, and the maximum treating pressure measured during the fracturing operations. A data set of 200 well production data and completion designs was collected from oil production wells in the Niobrara shale formation. Artificial neural network (ANN) and random forest (RF) techniques were implemented to predict EUR from the completion design. The results showed a low accuracy of direct prediction of the EUR from the completion design. Hence, an intermediate step of estimating the initial well production rate (*Q*_*i*_) from the completion data was carried out, and then, the *Q*_*i*_ and the completion design were used as input parameters to predict the EUR. The ANN and RF models accurately predicted the EUR from the completion design data and the estimated *Q*_*i*_. The correlation coefficient (*R*) values between actual EUR and predicted EUR from the ANN model were 0.96 and 0.95 compared with 0.99 and 0.95 from the RF model for training and testing, respectively. A new correlation was developed based on the weight and biases from the optimized ANN model with an *R* value of 0.95. This study provides ML application with an empirical correlation to predict the EUR from the completion design parameters at an early time without the need for complex numerical simulation analysis. The developed models require only the initial flow rate along with the completion design to predict EUR with high certainty without the need for several months of production similar to the DCA models.

## 1. Introduction

In shale gas reservoirs, the ultralow permeability matrix is not capable to flow fluid at a feasible rate and delivering an acceptable drainage volume. Horizontal drilling with multistage fracture completion has turned out to be the key stimulation technology for the development of shale plays [1–3]. Wells are to accomplish a series of fracturing processes, with a high injection rate, large fracturing slurry volume, and low proppant concentration, during the multistage design [4].

The economic feasibility and production improvement of an oil and gas well largely depend on the efficiency of hydraulically generated fractures. Reserve estimation is the key step for economic and investment calculations. Reserve, estimated ultimate recovery (EUR), is the estimation of oil and gas volume that can be economically extracted under the current technological constrictions. Estimating EUR in very tight reservoirs and shale plays has long been challenging. Reserve assessment is a process that regularly updated the age of the reservoir production history. The data availability and the forecasting method are the two vital elements that determine the estimated EUR accuracy [5]. Therefore, the development strategies are highly dependent on the accuracy of the forecast. The high-confidence EUR estimate is the total hydrocarbon recovery when the well reaches the abandonment conditions. However, no development action is required. Hence, earlier and more accurate estimation of EUR is required for the field development.

Several methods can be used to evaluate EUR in the oil and gas reservoirs. These methods may be purely based on physics, and other methods are built on empirical and analogy methods. Each technique has its limitations and inaccuracies [6]. These techniques include analogy theory, volumetric calculations, material balance, rate transient analysis (RTA), decline curve analysis (DCA), type curves, and numerical simulation.

Volumetric calculations and analogy methods depend on knowing the reservoir dimensions and petrophysical properties, which are difficult to be estimated in tight formations and early time development [5, 7]. Similarly, material balance (MBE) techniques are based on PVT data to calculate hydrocarbon in place and estimate EUR. However, MBE requires extended production data in addition to accurate reservoir pressure measurements. Moreover, MBE has many assumptions, which makes its applicability in unconventional reservoirs unsatisfactory. RTA is an analytical or numerical method widely used for the production forecast of unconventional reservoirs [8–10]. However, RTA methods face drawbacks due to a lack of precise measurements of reservoir rock and fluid properties and appropriate awareness of the physics controlling multiphase flow conditions.

Numerical simulation and history matching techniques can be used to estimate the future well production and EUR. However, an accurate formation of petrophysical properties and fracture parameters is required, in addition to extended production data to be matched [7, 11–14].

The decline curve is the most commonly used technique for estimating the hydrocarbon EUR for its simplicity and low input parameters [15]. Arps' decline method [16] is the famous empirical correlation that has been generally used as the main industry model. However, Arp's method over-forecasts reserves when applied in tight permeability reservoirs [17, 18]. Several DCA models have been introduced to forecast production tailored for unconventional wells. A common method is the stretched exponential production decline (SEPD) [19], in addition to the Arps hyperbolic decline with a “best-fit” hyperbolic decline exponent “*b*” value, but all are based on empirical observations of a particular scenario and have their own limitations, which can yield unreasonable EUR estimation [15, 19–22].

Machine learning (ML) has been used for diverse applications in oil and gas and environmental problems. Different ML tools such as artificial neural network (ANN), random forest (RF), function networks (FNs), adaptive neuro-fuzzy inference system (ANFIS), and support vector machine (SVM) can be applied to predict specific parameters from readily accessible data [6, 23–26].

ANN machine learning method includes three main layer types. These can be defined as input and output layers, in addition to hidden layers. The input layer includes the input parameters that are handled by neurons within the hidden layers to finally calculate the output layer. The layers are linked with a set of weights and biases, which are boosted by many training processes. These weights and biases can be modified to ultimately accomplish the lowest achievable error in the objective [27]. ANN has been applied to build predictive models in different areas [28–31].

RF technique includes many decision trees (DTs) that attain great performance in a low-dimensional data set. In RF, many trees are structured together to overcome the overfitting problem in the single DT technique by adjusting different hyper-parameters to improve the model accuracy [32].

The completion design greatly influences the multistage fractured horizontal shale well production rates and estimated ultimate recovery (EUR). EUR estimation is a critical process to evaluate the well profitability. EUR can be estimated through different methods including analogy, volumetric, RTA, DCA, and numerical simulation. However, these techniques are either highly inaccurate or very complex and time-consuming processes. Therefore, this study emphasizes developing a new methodology to estimate EUR for multistage fractured horizontal shale wells in the Niobrara formation. The well-completion data were used as an input to forecast future production. Moreover, this study provides ML application with an empirical correlation to predict the EUR from the completion design parameters at an early time without the need for complex numerical simulation analysis. Unlike the available empirical DCA models that require several months of production to build a sound prediction of EUR, the ML models in this study require only the initial flow rate along with the completion design to predict EUR with high certainty.

## 2. Methodology

A data set of production data and completion design was collected, and points were collected from around 200 horizontal wells completed in Niobrara shale formations. These wells reached the abandonment conditions. Hence, EUR for each well is basically the total production until the abandonment conditions. Only these wells were selected for this study, so there is no need for the use of any method to estimate the EUR. Moreover, the initial production rate per month was recorded for each well. The data set includes the completion design parameters such as the lateral length, the number of stages, the total injected proppant and slurry volumes, and the maximum treating pressure measured during the fracturing operations.  Table 1 reviews the different statistical parameters for the data set to define the data position and range, in addition to the distribution shape. The ranges of the parameters are as follows: the lateral length of 1500–11200 ft, the number of stages of 5–62, and the corresponding EUR that varied from 1.2*E*4 to 3.9*E*5 BOE.  Figure 1 shows a matrix plot for the collected data set to present the connections between the input completion parameters and the EUR. The diagonal displays the spreading of the data and their ranges.

Pearson's (*R*) and Spearman's rank (RR) correlation coefficients were used to describe the relationship between the input and the output parameters. The two coefficients were calculated using the following equations.

(1) $$\begin{array}{c} RR=\frac{\left[\sum \left(Rx_{i}-\mu_{Rx}\right)\left(Ry_{i}-\mu_{Ry}\right)/n-1\right]}{\sigma_{Rx}\sigma_{Ry}}, \end{array}$$

(2) $$\begin{array}{c} R=\frac{\left[\sum \left(x_{i}-\mu_{x}\right)\left(y_{i}-\mu_{y}\right)/n-1\right]}{\sigma_{x}\sigma_{y}}, \end{array}$$

where RR is Spearman's rank correlation coefficients between the rank of output parameter (output = CA) and rank of the input parameters. *x*_*i*_ is the independent feature, which involves the lateral length, the number of stages, the total injected proppant and slurry volumes, and the maximum treating pressure measured during the fracturing operations, and *y*_*i*_ is the dependent parameter (CA). *μ*_*x*_, *μ*_*y*_, and*σ*_*Rx*_, *σ*_*y*_ are the mean and the standard deviation subscription. RR reflects the rank correlation coefficient, where the correlation coefficient is calculated for the index of the data instead of the actual variable values.

Figure 2 presents a heat map for Pearson's and Spearman's correlation coefficients between all the input features with each other and with the EUR. Pearson's and Spearman's correlation coefficients almost show the same value for the coefficient, which reflects no outlier effect on the data. Generally, the correlation coefficient varies from −1 to 1. At the correlation coefficient of −1, the EUR is a strong inverse related to the completion parameter. For the correlation coefficient of 1, a strong direct relationship is found between the EUR and the completion parameter. A strong relationship was found between the EUR and the initial flow rate with a correlation coefficient of 0.81. In addition, strong relation was found between the EUR and the well length and the number of stages with correlation coefficient higher than 0.5. Most of the parameters—correlation coefficient of at least 0.5 between the different completion parameters and EUR except the maximum treating pressure—showed correlation coefficient of 0.23.

### 2.1. Model Development

ANN and RF ML tools were implemented to the collected data set to forecast the EUR. For both techniques, the data set (200 data points) was used to build the model after optimizing the splitting ratio of the training to testing data sets. The quality of the model was measured using absolute average error (AAPE), which represents the error between the actual EUR from the well production data and the estimated values of EUR from the ML model. AAPE can be calculated as follows:

(3) $$\begin{array}{c} \text{AAPE}=\frac{\sum_{i=1}^{N}\left(y_{i\text{ actual}}-y_{i\text{ predicted}}/y_{i\text{ actual}}\right)\times 100\%}{N}, \end{array}$$

where *y*_*i* actual_ and *y*_*i* predicted_ are the actual and the estimated output values (EURs), respectively, and N is the number of points in the data set. The correlation coefficient (*R*) was used as the goodness-of-fit indicator between the actual EUR from the well production data and the estimated EUR value from the model, and it was calculated using equation (2), where *x*_*i*_ and *y*_*i*_ are the actual and the estimated EUR values, respectively.

Figure 3 presents a schematic for the different model developing processes. After data collection and transformation, the data sets were applied to train and test the ML models. Different training/testing ratios were tested for the training set to be from 70 to 90%. Meanwhile, ML hyper-parameters were tested to optimize the model performance. The hyper-parameters for ANN and RF are included in Table 2. Table 2 reviews the different hyper-parameters that were used to improve the ML models and the optimum option.

### 2.2. RF Model Results

RF module was implemented on the well-completion input parameters to calculate the EUR. The completion data include the perforation interval, number of stages, total proppant volume, total fluid volume, maximum treatment pressure, and the true vertical depth. Different RF hyper-parameters were tested to achieve the highest prediction accuracy. The optimized training/testing ratio was found to be 70/30%.  Figure 4 shows the actual versus the predicted EUR values. The model shows high accuracy during the training data set with *R* values between the actual and predicted EUR values of 0.93 and *R*^2^ of 0.85. The model accuracy lowered in the case of the testing data set with *R* of 0.79 and *R*^2^ of 0.63. These results reflect the underfitting problem, and there is a need for adding other input features for the model development. Hence, the initial flow rate was required to be added to the input features similar to most of the DCA tools where the *Q*_*i*_ is an essential parameter for the EUR prediction.

Therefore, an intermediate step of predicting the *Q*_*i*_ from the completion data was introduced. The predicted *Q*_*i*_ was then used as an input for the EUR prediction model. For the *Q*_*i*_ model, the optimum parameters for RF models were maximum features = “SQRT,” maximum depth = 20, and the number of estimators = 150.  Figure 5(a) presents the RF cross-plot in both training and testing sets for the *Q*_*i*_ model with perfect alignment with the 45-degree line. The RF model was able to predict the *Q*_*i*_ with *R* values of 0.98 and 0.95 for both training and testing data sets, respectively, and the AAPE was estimated to be 7%.

The predicted *Q*_*i*_ was used as an input in addition to the completion data to the RF model to predict the EUR. Similar to the *Q*_*i*_ model, the hyper-parameters were updated to reach the best model performance with maximum features = “auto,” maximum depth = 30, and the number of estimators = 100.  Figure 5(b) presents the RF cross-plot in both training and testing sets for the EUR model with perfect alignment with the 45-degree line. The RF model was able to predict the EUR with R values of 0.99 and 0.93 for training and testing data sets, respectively.

After model development, it is important to use the residual plot to inspect the assumptions of the least-squares regression. Consequently, the residuals were estimated by subtracting the calculated EUR from the actual values.  Figure 6 shows the distribution of the residuals, where the residual is randomly scattered around zero. The residuals follow the normal distribution, which displays that the scattering degree of the points is similar for all fitted EURs with no biases towered at the high or the low end of the EUR range.

### 2.3. ANN Model Results

Similar to the RF model, the ANN technique was implemented on the collected data points to develop the ANN model. The optimized hyper-parameters were designated based on the best model performance indicators. The ANN model was built with one hidden layer with 8 neurons. The “trainlm” function was selected to be the training function with “logsig” as the data transfer function.  Figure 7 presents the actual EUR values versus the estimated EUR cross-plot from the ANN model in training and testing data sets.  Figure 7 shows the capability of the ANN model to calculate the EUR as a function of completion data and initial flow rate with a good alignment with the 45-degree line. The R value for the training set was found to be 0.96 with an AAPE error of 13%. The testing data result in AAPE of 12% with *R* values of 0.12.

Similar to RF mode, the model regression was tested with the residual plot in Figure 8.  Figure 8(b) displays that residuals have a normal distribution with a mean value of zero, which displays that the varying degree of the data is similar for all matched EURs with no biases towered the high or the low end of the EUR array.

### 2.4. EUR-ANN Empirical Correlation

One of the main results of the study was the construction of a correlation to calculate the EUR without running the ANN module. The equation was built using the weights and the biases from the developed ANN model including one hidden layer, 8 neurons, and the transformation function of “logsig.” The following equation presents the developed correlation using the weights and biases:

(4) $$\begin{array}{c} \text{EUR}=\left[\sum_{i=1}^{n}W2_{i}\left(\frac{1}{1+e^{-{\left(W1_{i,1}x_{1}+W1_{i,2}x_{2}+W1_{i,3}x_{3}+W1_{i,4}x_{4}+W1_{i,5}x_{5}+W1_{i,6}x_{6}+W1_{i,7}x_{7}+b1_{i}\right)}^{2}}}\right)\right]+b_{2}, \end{array}$$

where *W*2_*i*_ is the weights for the neurons from the hidden layer to the output layer and its bias is *b*_2_. *W*1_*i*,1−7_ is the weights for the neurons from the input layer to the hidden layer for the input parameters (x_1-7_); the number of stages, the lateral length, the total injected proppant and slurry volumes, the maximum treating pressure measured during the fracturing operations, and the initial production rate and *b*1_*i*_ are the improved biases for the hidden layer related to each neuron (*i*) from 1 to neuron number (*n*) = 8. This equation was established based on the modified weights and biases of the optimized ANN model. The tuned weights and biases of the EUR model are recorded in Table 3 to be a substitute for equation (4).

In addition to the correlation coefficient between each input and the output parameters, a sensitivity analysis was conducted to examine the influence of each input on the model performance.  Table 4 summarizes the *R* value for the model for different cases with ignoring one parameter each time. The results agreed with the correlation coefficient results in Figure 2. The highest influenced parameter was found to be the lateral length and the number of stages, while the least affecting parameter was found to be the maximum treating pressure.

The literature showed different empirical and data-driven models to predict the EUR for unconventional reservoirs.  Table 5 summarizes the used machine learning models, numbers of input data, and the average error for the developed models. This study presents a superior performance with a smaller number of inputs. In addition, the main advantage of this study is the independence of the EUR estimation on the availability of the one-year production history.

## 3. Conclusions

This work presents the application of ANN and RF approaches to estimate the EUR of hydraulically fractured horizontal wells in the Niobrara shale formation as a function of the completion parameters such as lateral length, the number of stages, total injected proppant and slurry volumes, and the maximum treating pressure measured during the fracturing operations. The following are the main findings:

- Using the initial production rate is essential for accurate EUR prediction.
- The *R* values between actual EUR and estimated EUR from the ANN and RF models were greater than 0.95.
- The EUR of the multistage fractured horizontal wells is highly dependent on the lateral length and the number of stages.

The developed machine learning models can be applied to accurately estimate the EUR at the early stage of the well without the need of conducting expensive and time-consuming numerical simulations or waiting until a very late stage of the well's life for decline curve analysis.

## Figures and Tables

**Figure 1:** Matrix plot of the different parameters with the diagonal shows the data frequency spreading.

**Figure 2:** Heat map for Pearson's and Spearman's rank correlation coefficients between the inputs and the outputs (EUR and *Q*_*i*_).

**Figure 3:** Processes of building the different ANN and RF models.

**Figure 4:** Actual EUR values versus the estimated values from the RF model without including *Q*_*i*_ in the input data for the training set and the testing data set.

**Figure 5:** Actual versus the estimated RF results for (a) *Q*_*i*_ model and (b) EUR model.

**Figure 6:** Residual distribution of the EUR predicted from RF-based model.

**Figure 7:** Actual versus calculated EUR plot for the ANN model in the case of (a) the training and (b) the testing data sets.

**Figure 8:** EUR residuals from ANN-based model. (a) Residuals vs. EUR and (b) the frequency of the residuals.

**Table 1:** Statistical analysis parameters for the used data set.

	Stage count	Horizontal length, ft	True vertical depth, ft	Max treatment pressure, psi	Tot. proppant vol., is	Tot. fluid vol., bbl	*Q*_*i*_, BOE/month	EUR, BOE
Mean	26	5681	6902	7155	4.6 *E* + 06	1.0 *E* + 05	12341	1.4 *E* + 05
Std	11	1930	394	1229	2.4 *E* + 06	5.3 *E* + 04	5358	8.1 *E* + 04
min	5	1530	5451	3467	9.5 *E* + 04	1.7 *E* + 04	950	1.2 *E* + 04
25%	18	4463	6743	6500	3.3 *E* + 06	6.1 *E* + 04	9633	8.1 *E* + 04
50%	20	4705	6945	7341	4.0 *E* + 06	7.7 *E* + 04	11604	1.3 *E* + 05
75%	34	6878	7119	8002	5.2 *E* + 06	1.4 *E* + 05	15064	1.9 *E* + 05
Max	62	11256	8331	9794	1.4 *E* + 07	2.8 *E* + 05	27527	3.9 *E* + 05

**Table 2:** Different options for improving the developed ANN and RF models.

Parameter	Available options	Optimum option	
		*Q*_*i*_ model	EUR model
ANN model			
Number of hidden layers	1–3	Single hidden layer	Single hidden layer
Number of neurons in each layer	5–40	8	8
Training/testing split ratio	70%–90%	(Training/testing) 70/30%	(Training/testing) 70/30%
Training algorithms	Trainlm, trainbfg, trainrp, trainscg, traincgb, traincgf, traincgp, trainoss, traingdx	“Trainbr”	“Trainbr”
Transfer function	Tansig, logsig, elliotsig, radbas, hardlim, satlin	“Logsig”	“Logsig”
Learning rate	0.01–0.9	0.05	0.05

RF			
Maximum features	[“Auto,” “sqrt,” “log2”]	sqrt	Auto
Maximum depth	[3, 4, 5, ..., 30]	20	30
Number of estimators	[3, 4, 5, ..., 150]	150	100

**Table 3:** Tuned weights and biases of the ANN-based EUR equation.

	*W*_i,j_									
*i*/*j*	1	2	3	4	5	6	7	*L*1	*b*2	*L*2
1	0.712	0.485	−1.821	2.462	0.197	−0.572	0.495	−1.005	0.266	−2.363
2	0.504	−1.456	−1.989	1.736	1.277	−0.242	−0.133	1.090	−1.876	
3	0.858	−0.226	−1.678	1.828	0.617	−1.666	1.248	−1.345	2.066	
4	−0.394	0.810	−1.411	−2.510	0.981	0.061	−0.695	0.932	1.484	
5	1.178	0.856	0.714	0.178	−0.086	−0.650	0.856	−0.240	−1.969	
6	−0.108	2.889	−0.208	−1.658	−0.485	−0.511	0.334	−0.493	−2.799	
7	1.259	0.689	−0.468	0.157	−0.729	−1.321	−1.259	0.164	2.304	
8	0.447	−0.034	−1.070	1.123	−0.639	−1.185	−0.711	−0.375	2.351	

**Table 4:** *R* value for the model for different cases with ignoring one parameter each time.

Inputs	*R* value
All inputs (lateral length, *n* of stages, the total injected proppant and slurry volumes, and the maximum treating pressure, vertical depth)	0.93
Ignore (*n* of stages)	0.77
Ignore (vertical depth)	0.8
Ignore (lateral length)	0.75
Ignore (proppant volume)	0.82
Ignore (slurry volume)	0.8
Ignore (maximum treating pressure)	0.88

**Table 5:** Comparison between current study and published work.

Paper	ML model	*No.* of inputs	Production history required	AAPE
[33]	Multilayer feedforward neural network (MLFNN)	16 input	Required 1-year production	21.9
[34]	Random forest (RF)	13 inputs		31%
[35]	Multiple linear regression model	19 geological and engineering factors	Required 1-year production	20%
[36]	Deep feedforward neural network algorithm	16 input	First-year average daily gas production	13–48%
Current study	ANN, RF	7 inputs	Initial production can be predicted as an intermediate step	7–12%

## Data Availability

Most of the data are available in the manuscript, and a detailed sample will be provided upon request.

## Nomenclatures

AAPE: Average absolute percentage error
ANN: Artificial neural network
N: Number of data points
ML: Machine learning
MLFNN: Multilayer feedforward neural network
R: Pearson's correlation coefficient
RR: Spearman's rank correlation coefficient
RF: Random forest
*x*_*i*_: Independent parameter
*y*_*i*_: Dependent parameters
*σ*_*x*_and*σ*_*y*_: Standard deviation for the independent and dependent parameters
*μ*_*x*_and*μ*_*y*_: Mean for the independent and dependent parameters
EUR: Estimated ultimate recovery
*Q*_*i*_: Initial production rate
BOE: Barrel of oil equivalent
*W*2_*i*_: Weights for the neurons from the hidden layer to the output layer and its bias is *b*_2_.
*W*1_*i*,1−7_: Weights for the neurons from the input layer to the hidden layer for the input parameters (*x*_1-7_)
*b*1_*i*_: Improved biases for the hidden layer related to each neuron (*i*) from 1 to neurons number (*n*) = 8.
